# Serum Levels of Mitochondrial Fission- and Fusion-Related Genes of Coal Workers' Pneumoconiosis and Risk Factor Analysis Based on a Generalized Linear Model

This article has been retracted.

**DOI:** 10.1155/2022/8629583

**Published:** 2022-04-01

**Authors:** Xiao-Yu Li, Jing-Lin Wei, Yong-Xin Xie, Ji Zhao, Li-Ya Ma, Na Zhang, Hui-Fang Yang

**Affiliations:** School of Public Healthy and Management, Key Laboratory of Environmental Factors and Chronic Disease Control, Ningxia Medical University, Yinchuan 750004, China

## Abstract

**Objective:**

We aimed to explore the risk factors for coal workers' pneumoconiosis and to further explore the significance of mitochondrial fission and fusion factors in CWP and verify the feasibility of mitochondrial fission and fusion factors as diagnostic and therapeutic targets.

**Methods:**

The data of 168 cases were collected, and they were divided into a healthy control group (40 cases), dust exposure control group (61 cases), and CWP group (67 cases) and entered into SPSS 24.0. The statistical data were analyzed by the chi-square test or Fisher's exact probability method. The variables with statistically significant differences of the univariate analysis results were included in the generalized linear model. Test level was *α* = 0.05. Blood samples were collected to detect the ROS content, MDA content, and SOD activity. The mRNA expression levels of *OPA1*, *Drp1*, *MFN2*, *Fis1*, *Col I*, *Col III*, and *α-SMA* were determined by q-PCR. The protein expression levels of OPA1, Drp1, MFN2, Fis1, Col I, Col III, and *α*-SMA were detected by western blot.

**Results:**

Generalized linear regression analysis showed that lower school education, no respiratory protective measures, the working age beyond 15 years, and the type of work like coal mine drillers were the risk factors for CWP. With the aggravation of CWP, the degree of fibrosis and inflammation increased oxidative damage, increased mitochondrion division, and decreased fusion, which were more sensitive in the second and third stages of CWP.

**Conclusion:**

The results in this found that mitochondria are injured by fission and fusion in the CWP patients. Detection of the mitochondria fission and fusion factors provides the application value to evaluate the injury degree and progress of CWP and the clues for finding the real and effective screening and diagnosis biomarkers.

## 1. Introduction

Coal remains an essential energy source worldwide; despite the global development of alternative energy sources, coal still accounts for nearly a third of global energy production [1], and coal dust is also a major pollutant causing environmental problems. Employment of mining industry will remain high for years, and contemporary miners will continue to face respiratory illnesses related to dust exposure. The disease is irreversible once the fibrosis occurs [2]. Pneumoconiosis is the most severe occupational disease worldwide, especially in developing countries, and the underlying mechanism has not been elucidated clearly [3].

In China, dust exposure in coal mining is one of the main occupational hazard factors. CWP (coal workers' pneumoconiosis) is one of the main types of 12 occupational pneumoconioses [4]. In recent years, the situation of occupational pneumoconiosis in China is not optimistic, and the incubation period of CWP is also increasing [5]. According to the Statistical Bulletin on the development of public health published by the National Health Commission of the People's Republic of China, the number of new cases of pneumoconiosis in 2017, 2018, and 2019 was 22701, 19468, and 15898, respectively; the proportion of the total number of newly reported occupational diseases was 84.84%, 82.85%, and 81.83%. At present, symptomatic treatment is mainly adopted to relieve the pain of patients. Therefore, it is crucial to explore the risk factors for pneumoconiosis and find the disease biomarkers [4, 6].

Pulmonary fibrosis is the most important manifestation of CWP, which is characterized by abnormal proliferation of fibroblasts and deposition of the extracellular matrix, leading to lung tissue damage eventually. The specific mechanisms mainly include direct cytotoxicity, imbalance of oxidative stress system, inflammatory response, proliferation of fibroblasts, and formation of pulmonary fibrosis [7].

In healthy individuals, mitochondrial division and fusion are kept in the relatively balanced state. On the one hand, mitochondrial fusion combines damaged mitochondria with healthy ones to produce elongated mitochondria, and the damaged part of the mitochondria combines with the healthy part as a complementary form to relieve the stress [5, 8]. On the other hand, mitochondrial division occurs after mitochondrial damage. If the stress persists, mitochondria will divide continuously and produce short and small fragments [9]. A tendency to increase mitochondrial fragmentation was also found in fibrosis models [10].

Regulatory proteins involved in mitochondrial fusion include OPA1 (optic atrophy 1), MFN1 (mitochondrial fusion protein 1), and MFN2 (mitochondrial fusion protein 2) [11]. OPA1 exists in the inner mitochondrial membrane (IMM), and it is a key substance in mitochondrial dynamics as well and interacts with other dyneins, including MFN1 and MFN2 which exist on the outer membrane of mitochondria [12]. The protein involved in mitochondrial division is dynamin-related protein 1 (Drp1), which exists in the cytoplasm; it can be recruited by Fis1 (mitochondrial fission protein 1) to form a spiral loop to induce mitochondrial division [13].

In recent years, mitochondrial mitotic fusion has become a research focus of fibrosis disease. In acute and chronic kidney disease, the imbalance of mitochondrial mitotic fusion will lead to mitochondrial dysfunction, kidney microvascular damage, inflammation, fibrosis, and kidney failure [14]. In animal experiments, targeted regulation of mitochondrial division and fusion could reverse the development of liver fibrosis [15]. In the model of idiopathic pulmonary fibrosis, an increase in abnormal morphology of mitochondria had also been found, and mitochondrial classification fusion disorder occurred [16].

In order to explore the role of mitochondrial fission and fusion factors in the occurrence and development of dust-induced pulmonary fibrosis, our research group established cell and animal coal workers' pneumoconiosis models in the early stage; the animal experiments have been submitted but have not yet been published. At present, the role of mitochondrial fission fusion factor in dust-induced pulmonary fibrosis has not been fully verified at the population level [17]. In order to propose targeted preventive measures, further explore the significance of mitochondrial fission-fusion factor in CWP and verify the feasibility of mitochondrial fission-fusion factor as a diagnostic and therapeutic target. We collected epidemiological survey data and blood samples from coal mine workers (healthy ones, dust-exposed ones, and workers with CWP). Through statistical analysis and laboratory testing, we focused on the following three questions:(1) risk factors for CWP occurrence, (2) the levels of fibrosis, inflammation, oxidative stress, and mitochondrial fission and fusion in the blood of coal workers' pneumoconiosis, and (3) whether the mitochondrial fission and fusion factor is correlated with the risk factors for coal workers' pneumoconiosis, fibrosis, inflammation, and oxidative stress levels. This study is aimed at exploring the effective diagnostic and therapeutic targets for CWP and providing new ideas for the treatment of CWP.

## 2. Methods

### 2.1. The Questionnaire Survey

In this study, inpatients admitted to Ningxia Occupational Hospital from December 2018 to May 2019 and employees of an occupational physical examination of a coal mine enterprise were enrolled, all of whom were males, 168 cases in total. They were divided into a healthy control group (40 cases), dust exposure control group (61 cases), and CWP group (67 cases). Medical records were verified for all patients included in this study, and the medical records are provided by the occupational disease hospital of Ningxia, including chest X-ray or chest CT changes. Among them, the healthy control group was white collar workers with nondust exposure in coal mines, the dust control group was people who engaged in coal mine-related work and had a definite history of dust exposure but were not diagnosed with CWP, and the CWP group was those who had a definite history of dust exposure and were diagnosed with CWP, including 12 cases in phase I, 29 cases in phase II, and 26 cases in phase III, and the medical records were subsequently checked one by one. All included study subjects gave informed consent.

#### 2.1.1. Inclusion Criteria

Healthy control group: males with no previous occupational exposure to dust and voluntary participation. Dust exposure control group: those with clear occupational exposure history but not diagnosed with coal workers' pneumoconiosis and voluntary participation. CWP group: patients with clear occupational exposure history, diagnosed by medical institutions with occupational disease diagnosis qualification, and pneumoconiosis classified as phases I, II, and III based on China's “Diagnosis of Occupational Pneumoconiosis” (GBZ 70-2015, http://www.samr.gov.cn/) and voluntary participation. The diagnosis of coal workers' pneumoconiosis was based on the history of exposure to coal dust and should be confirmed by chest X-ray or chest CT changes. All cases' medical records were verified.

#### 2.1.2. Exclusion Criteria

The exclusion criteria include patients with fibrosis diseases of other organs (such as the heart, liver, and kidney) and patients with pulmonary fibrosis caused by nondust factors.

### 2.2. Epidemiological Investigation

The epidemiological questionnaire was designed by the expert group of Ningxia Medical University, and the preliminary survey was conducted before the formal survey to understand the overall situation after the full implementation. The questionnaire was designed to collect information on the general condition of the study subjects (name, birth year, and education level), characteristics of individual behavioral factors (smoking situation, drinking situation), and characteristics of occupational factors (job type, dust working age, day working time, and whether respiratory protective measures were available during the operation). The investigators conducted face-to-face interviews with study subjects; then, the data were uniformly entered into the computer system by the investigators. Our study was based on patients' epidemiological survey and blood sample analysis. The research objects of this research were coal workers' pneumoconiosis patients who had clear history and healthy controls and dust exposure controls; the main research index such as oxidative stress, inflammation, and fibrosis index and serum sample would be more appropriate for research. Therefore, sputum was not collected.

### 2.3. Definitions of Variables

1. Dust exposure working age: the time from initial dust exposure to completely free from dust operation time
2. Job type: workers' job position. According to the work level, the work categories of coal miners were divided into coal mine drillers, coal miners, and auxiliary workers. Coal mine drillers mainly worked at the rock level and are exposed to rock dust; coal miners were mainly exposed to coal dust when working in coal beds, but some were also exposed to rock dust; and the auxiliary workers were mainly responsible for maintenance, transportation, and electric and mechanical equipment area

### 2.4. Data Collection and Statistical Analysis Methods

Data were collected and entered into Microsoft Excel 2019, and SPSS 24.0 statistical software was used for analysis. The statistical data were analyzed by the chi-square test or Fisher's exact probability method. Pairwise comparisons of count data were performed by the Bonferroni method. The variables with statistically significant differences of the univariate analysis results were included in the generalized linear model, and the 95% CI and *P* value were calculated. The experimental data were compared between multiple groups by one-way ANOVA and pairwise comparison by LSD. The Kruskal-Wallis *H* test was used for intergroup comparison of data that did not meet the nonparametric test. The test level was *α* = 0.05. The experimental data were performed into histograms by using GraphPad Prism 8.4.

### 2.5. Quality Control

To ensure the quality of the questionnaires, 2-3 postgraduate students from public health professions were selected to carry out the survey each time when they conducted the questionnaires. All the investigators learned relevant expertise of the questionnaires before conducting epidemiological surveys.

### 2.6. Data Entry Quality Control

After each data collection, the graduate students who participated in the survey on the same day input the data together and conducted a second check after completion.

### 2.7. Laboratory Detection

#### 2.7.1. Chemicals

Serum protein extraction kit (BB-319926, BestBio Science, Shanghai, China), Human ROS (reactive oxygen species) enzyme-linked immunoassay (Huijia Biotechnology Co., Ltd., Xiamen, China), SOD (superoxide dismutase) assay kit, and MDA (malondialdehyde) assay kit (A001-3-2, A003-1-2, Nanjing Jiancheng Bioengineering Institute, Nanjing, China) were used. Rabbit anti-MFN2 polyclonal antibody (sc-515647, Santa Cruz Biotechnology, Inc. USA), rabbit anti-Drp1 polyclonal antibody (8570S, Santa Cruz Biotechnology, Inc. USA), rabbit anti-OPA1 polyclonal antibody (67589S, Santa Cruz Biotechnology, Inc. USA), rabbit anti-Fis1 polyclonal antibody (sc-376446, Santa Cruz Biotechnology, Inc., USA), Rabbit anti-Col I (collagen type I) polyclonal antibody (AF7001, Affinity Biosciences, Inc., Jiangsu, China), rabbit anti-Col III (collagen type III) polyclonal antibody (AF0136, Affinity Biosciences, Inc., Jiangsu, China), rabbit anti-*α*-SMA (*α*-smooth muscle actin) polyclonal antibody (ab5694, Abcam Biotechnology, Inc., USA), and goat anti-rabbit IgG-HRP and goat anti-mouse IgG-HRP (ZB-2301, ZB-2305, Beijing Zhongshanjinqiao Biotechnology Co., Ltd., Beijing, China) were utilized.

#### 2.7.2. Blood Sample Collection and Pretreatment

3-5 mL venous blood of subjects of the healthy control group, dust exposure control group, and CWP group was collected and stored temporarily in a foam chamber at low temperature. After taking it back to the laboratory, it was centrifuged at 12000 × *g* for 10 min at 4°C. The upper transparent liquid was the serum sample, and each serum sample was divided into 3 parts, about 400 *μ*L for each, and then stored in the refrigerator at -80°C for standby application, avoiding repeated freeze-thaw cycles.

#### 2.7.3. Determination of ROS Content

The ROS content of human serum was determined by enzyme-linked immunoassay (ELISA), the OD (optical density) of the sample was measured at 450 nm, and the OD value of the sample was obtained by comparing the absorbance value of the blank hole; the measured standard OD value and the corresponding concentration were taken as the ordinate and abscissa, respectively, to draw the standard curve and get the regression equation. According to the OD value, the corresponding concentration of each sample was calculated. All measurements were performed at least in triplicate.

#### 2.7.4. Determination of Human Serum MDA Content

The content of MDA in serum was determined by the TBA method. The absorbance was measured at 532 nm; according to the OD value, the corresponding concentration of each sample was calculated. The final concentration was expressed as nmol/mL. MDA content (nmol/mL) was calculated as follows:

(1) $$\begin{array}{c} \text{MDA contents}=\frac{\text{O}{\text{D}}_{\text{sample value}}-\text{O}{\text{D}}_{\text{control value}}}{\text{O}{\text{D}}_{\text{standard value}}-\text{O}{\text{D}}_{\text{blank value}}}\times \text{Standard concentration}\times \text{Dilution ratio of sample}. \end{array}$$

#### 2.7.5. Determination of Human Serum SOD Activity

SOD activity of human serum was determined by the WST-1 method, and the absorbance value was measured at 450 nm; according to the OD value, the corresponding concentration of each sample was calculated, and the final concentration was expressed as U/mg protein. The SOD activity value (U/mL) was calculated as follows:

(2) $$\begin{array}{c} \text{SOD activity}=\text{supression ratio}÷50\%\times \left(\frac{0.24\text{mL}}{0.02\text{mL}}\right)\times \text{Dilution ratio of sample}. \end{array}$$

#### 2.7.6. qPCR

The expression of human serum genes was determined by quantitative real-time PCR (qPCR). Total RNA was extracted by using the Trizol reagent. GAPDH was used as an endogenous control and for normalization of gene targets. The primer sequences are shown in Table 1. Three multiple holes were detected in each sample, and the results of qPCR were quantitatively analyzed by 2^−ΔΔCt^. All assays were performed in triplicate.

#### 2.7.7. Determination of Protein Expression Level of Human Serum by Western Blot

The proteins (20 *μ*g/lane) were separated by 10% SDS-polyacrylamide gel electrophoresis and electrotransferred onto PVDF membranes. After being blocked with 3% BSA and incubated overnight at 4°C with a primary antibody against OPA1, Drp1, MFN2, Fis1, Col I, Col III, and *α*-SMA, then secondary antibodies were incubated. Bands were detected by using an ECL kit and the Invitrogen iBright 1500 Imaging System. Quantification of the western blot data was performed by using ImageJ software. Each experiment was repeated at least three times.

## 3. Results

### 3.1. Analysis of General Demographic Characteristics of Coal Workers

In this study, a total of 168 coal workers (40 from the healthy control group, 61 from the dust exposure control group, and 67 from the CWP group) were collected and analyzed for the basic demographic characteristics of the three groups. The results showed that the overall educational level composition were not the same (all *P* < 0.05). The pairwise comparison showed that there were more people over 70 years old (70~) in the CWP group (*P* < 0.05). Patients in the CWP group were generally less educated and mainly had primary school education or below, which were significantly different from those of healthy controls and dust-exposed controls, respectively (all *P* < 0.05) (Table 2).

### 3.2. Analysis on the Characteristics of Individual Behavior Factors of Coal Workers

The behavioral factors (smoking and drinking) that may affect the incidence of pneumoconiosis were analyzed. The chi-square test showed that there was no statistical significance in smoking, smoking index, drinking, or drinking index among the three groups (*P* > 0.05) (Table 3).

### 3.3. Analysis of Characteristics of Occupational Factors

The characteristics of occupational factors were analyzed in terms of daily working hours, dust exposure years, and types of work. The CWP group and dust exposure control group were divided into two groups according to working hours (h): <8 h and ≥8 h. The daily working time of most dust exposure control group was less than 8 h. *χ*^2^ test results showed that there was a statistically significant difference in the composition of working hours in the CWP group compared with the dust exposure control group (*P* < 0.05).

The CWP group and dust exposure control group were merged into one and then divided into two groups according to the work duration years of dust exposure (<15 years and ≥15 years). The results showed that the work duration years of dust exposure were related to the CWP disease (*P* < 0.05). It is suggested that the longer the dust exposure time, the greater the possibility of the CWP disease. Then, according to different positions, three groups were regrouped as the coal mine drillers' group, the coal miners' group, and the auxiliary workers' group; the results showed that the overall composition ratios were different (*P* < 0.05). Workers with or without respiratory protective measures were also shown to have the difference in these two groups (*P* < 0.05) (Table 4).

### 3.4. Multivariate Analysis of Risk Factors for Coal Workers' Pneumoconiosis

According to the results of the *χ*^2^ test, 5 variables with statistical differences (degree of education, respiratory protective measures, type of position, working hours, and work duration years) were included into the generalized linear model, and the factors affecting the occurrence of CWP were analyzed.

The results of the generalized linear regression analysis showed that, in terms of educational attainment, “primary school and below” was considered the reference and “junior high school and above” was a protective factor for CWP (*B* = 3.475, 95%CI = 1.762~5.187). In terms of respiratory protective measures, “no respiratory protective measure” was considered a reference and “having respiratory protective measures” was a protective factor for CWP (*B* = −2.151, 95%CI = −3.710 ~ −0.592). In terms of work duration years, “work duration years < 15” was considered a reference and “work duration years ≥ 15” was a risk factor for CWP (*B* = −2.086, 95%CI = −3.779 ~ −0.392). In terms of working positions, “auxiliary workers” was considered a reference and “coal mine drillers” was a risk factor for CWP (*B* = 1.654, 95%CI = 0.316 ~ 3.319) (Tables 5 and 6).

### 3.5. Expression of Fibrosis Genes in Serum

Compared with the healthy control group, the relative mRNA expression levels of *Col I* and *Col III* and *α-SMA* in the blood samples of 4 groups (dust exposure control group and CWP phase I, II, and III groups) were increased, and the differences were statistically significant (*F* = 103.9, 70.67, and 161.05, *P* < 0.05). Further pair comparison showed that, compared with the healthy control group, the relative mRNA expression levels of *Col I* and *Col III* in CWP phase II and III groups were increased, and the relative expression levels of *α-SMA* mRNA in CWP I, II, and III groups were increased (*P* < 0.05). Compared with the dust exposure control group, the relative mRNA expression levels of *Col I* and *Col III* in CWP phase II and phase III groups were increased, and the relative mRNA expression levels of *α-SMA* in CWP phase I, II, and III groups were increased (*P* < 0.05) (Figure 1). Western blot analysis showed that, compared with the healthy control group, the relative protein expression levels of Col I, Col III, and *α*-SMA in CWP phase I, II, and III groups were increased (*P* < 0.05). Compared with the dust exposure control group, the relative protein expression levels of Col I and Col III in CWP phase II and III groups were gradually increased (*P* < 0.05), while the relative protein expression levels of *α*-SMA were gradually increased in CWP phase I, II, and III groups (*P* < 0.05) (Figure 2).

### 3.6. Expression of Inflammation-Related Genes in Serum

The differences of relative expression levels of *TNF-α* and *IL-6* mRNA in blood samples of all groups (healthy control group, dust exposure control group, and CWP phase I, II, and III groups) were statistically significant (*F* = 58.22 and 49.08, *P* < 0.05). Compared with the healthy control group, the relative expression levels of *TNF-α* and *IL-6* mRNA in CWP phase II and III groups were increased (*P* < 0.05). Compared with the dust exposure control group, the relative mRNA expression levels of *TNF-α* and *IL-6* in CWP phase II and III groups were increased (*P* < 0.05) (Figure 3).

### 3.7. Determination of Oxidative Stress Index in Serum

The ROS content of all groups (healthy control group, dust exposure control group, and CWP phase II and III groups) had an increased trend (*F*/*H* = 16.88, *P* < 0.05). The SOD activity of all groups had a decreased trend (*F*/*H* = 5.73, *P* < 0.05). The MDA content of all groups had an increased trend (*F*/*H* = 12.22, *P* < 0.05). And the relative mRNA expression levels of NOX2 in the blood samples of these groups were increased, and the difference was statistically significant (*F*/*H* = 38.91, *P* < 0.05). The results of further pairwise comparison showed that compared with the healthy control group, ROS content in CWP phase II and III groups was increased (*P* < 0.05), SOD activity in CWP phase I, II, and III groups was decreased (*P* < 0.05), the content of MDA in CWP phase II and III groups was increased (*P* < 0.05), and the relative expression of NOX2 mRNA in the CWP phase III group was increased (*P* < 0.05). Compared with the dust exposure control group, ROS content in the CWP phase II group was increased (*P* < 0.05), SOD activity in CWP phase II and III groups was decreased (*P* < 0.05), the content of MDA in CWP phase II and III groups was increased (*P* < 0.05), and the relative mRNA expression of NOX2 in CWP phase II and III groups was increased (*P* < 0.05) (Figure 4).

### 3.8. Expression of Mitochondrial Fission- and Fusion-Related Genes and Proteins in Serum

Western blot analysis showed that, compared with the healthy control group, the relative protein expression levels of OPA1 and MFN2 in CWP phase I, II, and III groups were increased (*P* < 0.05) and the relative expression levels of Fis1 and Drp1 were gradually decreased (*P* < 0.05). Compared with the dust exposure control group, the relative protein expression levels of OPA1 and MFN2 in CWP phase I, II, and III groups were gradually increased (*P* < 0.05), while the relative protein expression levels of Fis1 and Drp1 were gradually decreased (*P* < 0.05) (Figure 5).

## 4. Discussion

The main pathogenic factor of CWP is inhalation of coal dust for a long term; however, the mechanism of disease occurrence and development in the human body is complex and uncertain, which limits the methods of diagnosis, intervention, and treatment [18]. Pulmonary fibrosis is a typical pathological feature of CWP. Previous studies have hypothesized in animal and cellular fibrosis models, such as signaling pathways and cytokines [19]. Sadly, biomarkers of population samples of CWP have not been systematically studied in China.

Pulmonary fibrosis is a typical pathological feature of CWP [20, 21]; some studies have shown that after the lung is stimulated by foreign dust, the inflammatory reaction first occurs, which is also an important inducement of fibrosis. In inflammatory response, tumor necrosis factor-*α* (TNF-*α*) can directly or indirectly promote the development of fibrosis [22], and the correlation of TNF-*α* gene polymorphism with genetic susceptibility of pneumoconiosis has been demonstrated [23]. Interleukin-6 (IL-6) is an important regulator of TNF-*α*. IL-6 has been shown to predict lung injury prior to pathological changes on X-ray [24]. Increasing evidences demonstrate that IL-6 plays a central role in the acute phase reaction and tissue inflammation. In this study, the expression of TNF-*α* and IL-6 gradually increased with the progression of the disease, which was consistent with the results of Qian et al. and Slavov et al. [22, 25], suggesting that TNF-*α* and IL-6 could be used as biological indicators to evaluate the efficacy and prognosis of CWP.

Previous studies have shown that the occurrence and development of pneumoconiosis are usually accompanied by exacerbation of pulmonary fibrosis and abnormal oxidative stress [26]. With the aggravation of the disease, mitochondrial repair ability decreases. Studies have shown that ROS plays a regulatory role in mitochondrial division and fusion, and the reduction of mitochondrial division will further increase the production of ROS, leading to the regulation disorder of mitochondrial division and fusion and the aggravation of mitochondrial damage [27]. On the other hand, chronic inflammation promotes the formation of ROS; a large number of ROS disrupt the original balance of oxidation and induce fibrosis [28]. In this study, it was found that the expression of *NOX2* mRNA in the CWP group was increased, and the change of ROS was consistent with it. Stimulation from the outside of the cell is conducted by ROS-producing systems located in or near the plasma membrane, such as NADPH oxidase (NOX) complexes. Recent studies have uncovered a unique biological mechanism by which activation of the NADPH oxidase 2 (NOX2) complex, a major source of reactive oxygen species (ROS), enhances the cross-presentation by antigen-presenting cells (APCs) [29].

Dust stimulates cells to produce a large number of ROS, which destroys the original balance of oxidation and antioxidant and induces the occurrence of fibrosis. Low concentration of ROS in a short time will increase stress resistance, and the defense function will be activated to neutralize the damage caused by oxidation; it will not cause too much damage to the body, but the opposite effect will be produced in a long time. To remove extra ROS, cells release SOD and MDA to deploy a defense system. MDA is a recognized lipid peroxidation marker [30], and the increased expression level of MDA in CWP population is consistent with the research by other scholars, indicating the aggravation of oxidative damage in the body [31]. SOD is the first line of defense against oxidative stress [32], and the expression level of SOD in the CWP population is decreased, suggesting that SOD may be decomposable in order to eliminate free radicals produced by redox.

Fibrosis is the final response of chronic injury, which is usually caused by massive cell apoptosis and necrosis and produces a large amount of extracellular matrix, and fibroblasts are the main cells that construct and maintain these extracellular matrices [33]. *Col I*, *Col III*, and *α-SMA* are different types of collagen secreted by fibroblasts and can be used as markers of fibroblast cell proliferation [34]. In this study, as the fibrosis gets worse, the relative mRNA and protein expression levels of Col I, Col III, and *α*-SMA were increased, which further demonstrated that Col I, Col III, and *α*-SMA are effective biomarkers of fibrosis disease.

Mitochondrial fission and fusion are important regulatory mechanisms in human physiological and pathological states, which also are the parts of mitochondrial quality control. Mitochondria maintain the normal function by constant fission and fusion and respond to the damage caused by inflammation and oxidative stress [35]. Both oxidative stress and inflammation can cause mitochondrial fission and fusion, while overstress inhibits the expression of MFN1 and MFN2, which are in the outer mitochondrial membrane, and OPA1 which is in the inner mitochondrial membrane, preventing the formation of a continuous mitochondrial chain. At the same time, Fis1 is activated to gather around mitochondria, and Drp1 is collected to the surface of mitochondria, resulting in mitochondrial fragmentation and repair ability impairment, mitochondrial failure to maintain normal homeostasis and dysfunction, cell apoptosis, activation of fibroblasts, and exacerbation of the disease [36]. Our study confirmed that the decreased expression level of mitochondrial fusion genes (*OPA1*, *MFN*2) and the increased expression level of mitochondrial division genes (*Drp1*, *Fis1*) in patients with coal workers' pneumoconiosis suggested that the number of short mitochondria increased, and the repair ability of damaged mitochondria decreased, resulting in cellular dysfunction.

It is generally believed that dust exposure time is positively correlated with dust exposure rate [37]; we divided the subjects into two groups: ≤15 years group and >15 years group, according to the work duration years of dust exposure. The results suggested that the longer the working age, the longer the dust exposure time and the higher the dust exposure rate is; thus, the occurrence and development of CWP will be promoted. In addition, studies have shown that the longer the exposure time, the higher the incidence of some complications, such as chronic obstructive pulmonary disease (COPD), tuberculosis, and cardiovascular and cerebrovascular diseases [38].

As bad living habits, smoking and drinking are considered to aggravate or promote the development of diseases to a certain extent; the results showed that there was no statistical significance in smoking, smoking index, drinking, or drinking index among the three groups; previous studies have shown similar results to our study [39]. The results of this study indicated that the absence of respiratory protection was also a risk factor for CWP, due to the increasing chance of dust entering the respiratory tract. The study showed that it was often difficult to reduce the dust of the air to a safe concentration in the control scheme of the production process, but respiratory protection could effectively prevent the dust from entering the respiratory tract, such as masks [32]. By taking the auxiliary workers as the reference, the work type like the coal mine drillers was the risk factor for CWP. According to the work level, the occupational types of coal miners are divided into coal mine drillers, coal miners, and auxiliary workers. The coal mine drillers mainly worked at the rock level and are exposed to rock dust, mainly composed of silica [40]. Therefore, the focus of comprehensive dust prevention in coal mine enterprises should be the coal mine drillers, and special protection should be carried out according to the type of work. Coal mine drillers are the focus of pneumoconiosis prevention and control work. In coal mine work, coal mine drillers and coal miners are frontline workers with the highest concentration of exposure to productive dust and a high possibility of developing CWP, which should reduce the number of years of exposure to dust, reduce the time workers are exposed to occupational hazards and delay the occurrence of CWP, strengthen health education for workers and establish a positive concept of life, and improve the awareness of workers' protection. The company needs to pay attention to the physical health condition of workers and conduct medical checkups on a regular basis. Workers with a relative high level of education have a high degree of recognition of risk factors in the work environment, so they may have a strong sense of self-protection. Therefore, enterprise leaders should attach great importance to workers' health and organize health education lectures before and during workers' employment, to help workers establish a positive life concept and strengthen their health awareness to prevent or delay the occurrence and development of CWP. Meanwhile, ventilation systems, water sprays, and other dust capturing devices should be in continuous usage, and ensure they are operating at an optimal level continuously [2].

With the aggravation of CWP, the degree of fibrosis, inflammation, and oxidative damage increased, the mitochondrial division increased and the fusion decreased, and all those indicators were more sensitive in the CWP II and III stage. The role of mitochondrial fission and fusion genes in the occurrence and development of CWP needs to be further studied by increasing the sample size.

## 5. Conclusion

The results in this found that mitochondria are injured by fission and fusion in the CWP patients. Detection of the mitochondria fission and fusion factors provides the application value to evaluate the injury degree and progress of CWP and the clues for finding the real and effective screening and diagnosis biomarkers.

## Figures and Tables

**Figure 1:** Relative expression level of fibrosis-related genes. (a) The relative mRNA expression levels of *Col I*. (b) The relative mRNA expression levels of *Col III*. (c) The relative mRNA expression levels of *α-SMA*. ^a^*P* < 0.05, compared with the healthy control group. ^b^*P* < 0.05, compared with dust exposure control group.

**Figure 2:** Relative expression level of fibrosis-related proteins by western blot analysis. (a) Expression of fibrosis-related proteins in serum by western blot analysis. (b) The relative protein expression level of Col III. (c) The relative protein expression levels of Col I. (d) The relative protein expression level of *α*-SMA. ^a^*P* < 0.05, compared with the healthy control group. ^b^*P* < 0.05, compared with the dust exposure control group.

**Figure 3:** Relative expression of TNF-*α* and IL-6 mRNA. (a) The relative mRNA expression levels of TNF-*α*. (b) The relative mRNA expression levels of IL-6. ^a^*P* < 0.05, compared with the healthy control group. ^b^*P* < 0.05, compared with the dust exposure control group.

**Figure 4:** Oxidative damage of coal workers' pneumoconiosis changes. (a) The ROS content of human serum samples. (b) The superoxide dismutase (SOD) activity of human serum samples. (c) The malondialdehyde (MDA) content of human serum samples. (d) The relative mRNA expression of *NOX2* in human serum samples. ^a^*P* < 0.05, compared with the healthy control group. ^b^*P* < 0.05, compared with the dust exposure control group.

**Figure 5:** Relative protein expression levels of fission- and fusion-related genes in serum of coal mine workers. (a) Expression of mitochondrial fission- and fusion-related genes and proteins in serum by western blot analysis. (b) The relative protein expression level of OPA1. (c) The relative protein expression level of Drp1. (d) The relative protein expression levels of MFN2. (e) The relative protein expression level of Fis1. ^a^*P* < 0.05, compared with the healthy control group. ^b^*P* < 0.05, compared with the dust exposure control group.

**Table 1:** Primers used for gene expression analysis by qPCR.

Gene name	NCBI reference sequence	Direction	Primer sequence (5′-3′)
*IL-6*	NM_000600.5	Forward	GGTGTTGCCTGCTGCCTTCC
		Reverse	GTTCTGAAGAGGTGAGTGGCTGTC
*TNF-α*	NM_000594.4	Forward	AAGGACACCATGAGCACTGAAAGC
		Reverse	AGGAAGGAGAAGAGGCTGAGGAAC
*α-SMA*	NM_001613.4	Forward	CTCTGGACGCACAACTGGCATC
		Reverse	CACGCTCAGCAGTAGTAACGAAGG
*COL III*	NM_000090.4	Forward	GTAACACTGGTGCTCCTGGC
		Reverse	ACCAGGCGATCCCTTCTCTC
*COL I*	NM_000088.4	Forward	GTGGTCAGGCTGGTGTGATG
		Reverse	GCCTTGTTCACCTCTCTCGC
*NOX2*	NM_000397.4	Forward	TTCCAGTGCGTGCTGCTCAAC
		Reverse	TGGTGTGAATCGCAGAGTGAAGTG

**Table 2:** Analysis of general demographic characteristics of workers in coal mining enterprises.

Demographic characteristic	Healthy control group, *n* (%)	Dust exposure control group, *n* (%)	CWP group, *n* (%)	*χ* ^2^/Fisher	*P* value
Age (year)					
<50	13 (32.5)	9 (14.8)	3 (4.5)	42.925	<0.001^∗^^#^
50~	22 (55.0)	42 (68.9)	25 (37.3)		
70~	5 (12.5)	10 (16.4)	39 (58.2)		
Educational level					
Primary school or below	4 (10.0)	7 (11.5)	52 (77.6)	76.529	<0.001^∗^^#^
Junior high school and above	36 (90.0)	54 (88.5)	15 (22.4)		
Marital status					
Married	40 (100.0)	59 (88.1)	60 (98.4)	10.977	<0.001^∗^^#^
Divorced or widowed	0 (0)	8 (11.9)	1 (1.6)		

Note: ^∗^*P* < 0.05 indicated that the difference was statistically significant compared with the healthy control group. ^#^*P* < 0.05 indicated that, compared with the dust exposure control group, the difference was statistically significant.

**Table 3:** Characteristic analysis of individual behavior factors of coal workers.

Individual behavior	Healthy control, *n* (%)	Dust exposure, *n* (%)	CWP group, *n* (%)	*χ* ^2^	*P* value
Smoking					
Yes	28 (70.0)	38 (62.3)	53 (79.1)	4.385	0.112
No	12 (30.0)	23 (37.7)	14 (20.9)		
Smoking index (pack-year)					
<30	27 (70.0)	55 (80.3)	53 (79.1)	2.566	0.277
≥30	13 (30.0)	12 (19.7)	8 (20.9)		
Drinking					
Yes	23 (57.5)	39 (63.9)	37 (55.2)	1.045	0.593
No	12 (30.0)	23 (37.7)	14 (20.9)		
Drinking index (L/year)					
<5	38 (95.0)	53 (86.9)	55 (82.1)	3.019	0.221
≥5	2 (5.0)	8 (13.1)	12 (17.9)		

**Table 4:** Analysis of occupational factor characteristics of coal workers.

Occupational factors	Dust exposure control group, *n* (%)	CWP group, *n* (%)	*χ* ^2^	*P* value
Working hours (h/d)				
<8	53 (86.9)	40 (59.7)	11.876	0.001^∗^
≥8	8 (13.1)	27 (40.3)		
Work duration (years/year)				
<15	28 (45.9)	5 (7.5)	24.656	<0.001^∗^
≥15	33 (54.1)	62 (92.5)		
Position				
Coal mine drillers	15 (24.6)	53 (79.1)	46.657	<0.001^∗^
Coal miners	10 (16.4)	10 (14.9)		
Auxiliary workers	36 (61.0)	4 (6.0)		
Respiratory protective measures				
Yes	36 (59.0)	20 (29.9)	11.037	<0.001^∗^
No	25 (40.1)	47 (70.1)		

Note: ^∗^*P* < 0.05 indicated that the difference was statistically significant.

**Table 5:** Generalized linear models analyze the assignment table.

Variable	Implication	Assignment instructions
X1	Degree of education	Primary school or below = 1, junior high school or above = 0
X2	Marital status	Married = 1, divorced = 0
X3	Respiratory protective measures	Have = 1, not have = 0
X4	Type of position	Coal mine drillers = 1, coal miners = 2, auxiliary workers = 0
X5	Working hours	≤8 = 1, >8 = 0
X6	Work duration years	<15 = 1, ≥15 = 0
*Y*	CWP	Have = 1, not have = 0

**Table 6:** Analysis of risk factors for coal workers' pneumoconiosis.

Variable	*B*	*S*_*b*_	Wald *χ*^2^	*P* value	95% CI
Educational level					
Primary school or below	3.372	0.9313	13.109	0.000^∗^	1.547~5.197
Junior high school and above	—	—	—	—	—
Marital status					
Married	-3.578	1.7911	3.991	0.046^∗^	-7.089~-0.068
Divorced or widowed	—	—	—	—	—
Respiratory protective measures					
Yes	-2.266	0.8441	7.210	0.007^∗^	-3.921~-0.612
No					
Working hours (h/d)					
≤8	-1.266	0.7408	2.921	0.087	-2.718~0.186
>8	—	—	—	—	—
Work duration (years/year)					
<15	-2.218	0.9416	5.547	0.019^∗^	-4.063~-0.372
≥15	—	—	—	—	—
Position					
Coal mine drillers	2.032	0.8598	5.583	0.018^∗^	0.346~3.717
Coal miners	-1.794	1.1502	2.433	0.119	-4.048~0.460
Auxiliary workers	—	—	—	—	—

## Data Availability

The data used to support the findings of this study are available from the corresponding author upon request.
